This article has been retracted.

# Phytomedicinal Role of *Pithecellobium dulce* against CCl_4_-mediated Hepatic Oxidative Impairments and Necrotic Cell Death

**DOI:** 10.1093/ecam/neq065

**Published:** 2011-03-13

**Authors:** Prasenjit Manna, Sudip Bhattacharyya, Joydeep Das, Jyotirmoy Ghosh, Parames C. Sil

**Affiliations:** Division of Molecular Medicine, Bose Institute, P-1/12, CIT Scheme VII M, Kolkata 700054, West Bengal, India

## Abstract

Present study investigates the beneficial role of the aqueous extract of the fruits of *Pithecellobium dulce* (AEPD) against carbon tetrachloride (CCl_4_)-induced hepatic injury using a murine model. AEPD has been found to possess free radical (DPPH, hydroxyl and superoxide) scavenging activity in cell-free system. CCl_4_ exposure increased the activities of various serum maker enzymes and intracellular reactive oxygen species (ROS) production. In line with these findings, we also observed that CCl_4_ intoxication increased the lipid peroxidation and protein carbonylation accompanied by decreased intracellular antioxidant defense, activity of cytochrome P450 and CYP2E1 expression. DNA fragmentation and flow cytometric analyses revealed that CCl_4_ exposure caused hepatic cell death mainly via the necrotic pathway. Treatment with AEPD both pre- and post-toxin exposure protected the organ from CCl_4_-induced hepatic damage. Histological findings also support our results. A well-known antioxidant vitamin C was included in this study to compare the antioxidant potency of AEPD. Combining all, results suggest that AEPD protects murine liver against CCl_4_-induced oxidative impairments probably via its antioxidative property.

## 1. Introduction

Liver diseases are a major problem throughout the world. Hepatic injury, induced by haloalkanes, has been recognized as one of the most common toxicological problems [1]. Carbon tetrachloride (CCl_4_), one of the chlorinated hydrocarbons, is widely used in various industries as a solvent. It is also used in medicine as a vermifuge in the treatment of hookworm disease. Exposure to CCl_4_ by inhalation, ingestion or absorption through the skin resulted in many cases of poisoning. In addition, CCl_4_ is used as a model for studying free-radical-induced liver injury and screening hepato-protective drugs [2]. Prolonged administration of CCl_4_ causes fibrosis, cirrhosis and hepatic carcinoma [3]. Emerging evidences indicate that oxidative stress might be a pivotal originating factor in the pathogenesis of CCl_4_-induced liver diseases [4, 5]. Although some of the basic mechanisms of free-radical reactions following CCl_4_ administration are largely known, a potential therapy against hepatotoxicity has not yet been achieved.

Numerous medicinal plants and their formulations are used for liver disorders in ethno-medical practice as well as traditional system of medicine in India [6, 7]. Plant products play a beneficial role in the management of various liver disorders [8–13]. In the absence of a reliable liver protective drug in the modern medicine, a number of medicinal preparations in ayurveda are recommended for the treatment of liver disorders. *Pithecellobium dulce* is a well-known Indian medicinal plant. *Pithecellobium dulce* has been commonly used for fencing and tanning, as fodder for feed and pods for food. Infusions of different parts of *P. dulce* have been traditionally used to treat diseases, for example, skin of the stem is used for dysentery, leaves for intestinal disorders and seeds for ulcers [14, 15].

Present study has been carried out to investigate the protective role of the aqueous extract of the fruits of *P. dulce* (AEPD) against CCl_4_-induced hepatic disorders. First, the radical scavenging activity of the extract was determined from its DPPH (1,1-diphenyl-2-picrylhydrazyl) radical quenching ability and the data were compared to those obtained from a known free-radical scavenger, vitamin C. Secondly, dose- and time-dependent studies have been conducted to evaluate the optimum conditions necessary for the extract to exhibit its maximum protective activity against CCl_4_-induced hepatic oxidative damages by measuring the levels of the serum marker enzymes, alanine transaminase (ALT) and alkaline phosphatase (ALP). The extent of hepatic damages caused by CCl_4_ and the protective role of AEPD was evaluated by measuring the (i) activities of intracellular antioxidant enzymes; (ii) the levels of cellular metabolites; (iii) the levels of lipid peroxidation, protein carbonylation (PC), intracellular reactive oxygen species (ROS) production and (iv) the activity of cytochrome P450 and the expression of its isoenzyme (CYP2E1). The mode of hepatic cell death has been evaluated by flow cytometry and DNA fragmentation analysis. In addition, histological studies were carried out to assess the ultrastructural changes in murine livers.

## 2. Methods

### 2.1. Plant

*Pithecellobium dulce*, one of the important medicinal plants of India, belongs to the family of Fabaceae. For this particular study, the fruits were collected in the summer season of the current year from the local market of Kolkata, India. After collection, one voucher specimen of this plant was deposited in the Central National Herbarium (CNH), Botanical Survey of India (BSI), Howrah, West Bengal, India.

### 2.2. Animals

All experiments were performed on Swiss albino mice (male, body weight 20 ± 2 g, purchased from M/S Gosh Enterprises, Kolkata, India.). The animals were acclimatized under laboratory conditions for 2 weeks prior to the experiments. They were maintained under standard conditions of temperature (23 ± 2°C) and humidity (50 ± 10%) with alternating 12 h light/dark cycles. The animals had free access to tap water and were fed standard pellet diet (Agro Corporation Private Ltd., Bangalore, India). The ethical committee of Bose Institute approved the guidelines of the experimental procedure using the animals (mice) and all the experiments with animals were carried out according to guidelines of the institutional animal ethical committee.

### 2.3. Chemicals and Other Reagents

Bradford reagent, DPPH, bovine serum albumin (BSA) and protein estimation kit were purchased from Sigma-Aldrich Chemical Company, (St. Louis, MO, USA). CCl_4_, disodium hydrogen phosphate (Na_2_HPO_4_), 1-chloro-2,4-dinitrobenzene (CDNB), 5,5′-dithiobis(2-nitrobenzoic acid) [DTNB, (Ellman's reagent)], ethylene diamine tetra acetic acid (EDTA), glacial acetic acid, hydrogen peroxide (H_2_O_2_), nicotinamide adenine dinucleotide reduced (NADH), sodium dihydrogen phosphate (NaH_2_PO_4_), nitro blue tetrazolium (NBT), phenazine methosulphate (PMT), reduced glutathione (GSH), sodium pyrophosphate, potassium dihydrogen phosphate (KH_2_PO_4_), trichloroacetic acid (TCA), thiobarbituric acid (TBA) were bought from Sisco Research Laboratory, India.

### 2.4. Aqueous Fruit Extract Preparation

After collection, the fruits were cut into small pieces and homogenized in 50 mM phosphate buffer, pH 7.2 at 4°C. The homogenized mixture was centrifuged at 12 000 g for 30 min to get rid of unwanted debris and lyophilized. The freeze-dried material was weighed, dissolved in the same phosphate buffer and used in different experiments needed for this study.

### 2.5. Qualitative Analysis of AEPD

Phytochemical analysis of AEPD was carried out to investigate the presence of active ingredients like flavonoids, saponins, phenolics, steroids, and so forth.

A portion of crude powder was heated with 10 ml of ethyl acetate over a steam bath for 3 min. The mixture was filtered and 4 ml of the filtrate was shaken with 1 ml of dilute ammonia solution. Appearance of yellow coloration confirmed the presence flavonoids in the extract [16].

To find out the presence of saponins, small amount (0.5 g) of crude powder was shaken with water in a test tube and it was warmed in a water bath. Persistent froth formation indicated the presence of saponins in the extract [17, 18].

About 0.5 g of crude powder was heated with 5 ml of ethyl alcohol over a steam bath for 3 min and then few drops of neutral ferric chloride solution were added. Appearance of violet coloration confirmed the presence phenolic compounds in the extract [19].

For the analysis steroid compounds, about 0.5 g of crude powder was dissolved in 5 ml of methanol. 1 ml of the alcoholic extract was treated with 0.5 ml of acetic anhydride and the solution was cooled in ice. The mixture was then mixed with 0.5 ml of chloroform and 1 ml of concentrated sulfuric acid [20]. A reddish-brown ring was formed at the separations level of the two liquids and appearance of this ring indicated of the presence of steroids in the extract.

### 2.6. Quantitative Analysis of AEPD

#### 2.6.1. Flavonoid Content Estimation

Ten grams of crude powder was extracted repeatedly with 100 ml of 80% aqueous methanol at room temperature. The whole solution was filtered through Whatman filter paper no. 42 (125 m). The filtrate was transferred into a crucible, evaporated into dryness and weighed to a constant weight [21].

#### 2.6.2. Determination of Saponin Content

Twenty grams of crude powder was put into a conical flask and 100 ml of 20% aqueous ethanol were added. The samples were heated over a hot water bath for 4 h with continuous stirring at about 55°C. The mixture was filtered and the residue was extracted with another 200 ml of 20% ethanol. The extract was reduced to 40 ml over water bath at about 90°C. The concentrate was transferred into 250 ml separating funnel, 20 ml of diethyl ether was added and the mixture was shaken vigorously. The aqueous layer was recovered while the ether layer was discarded. The purification process was repeated. An amount of 60 ml of *n*-butanol was then added. The combined *n*-butanol extracts were washed twice with 10 ml of 5% aqueous sodium chloride. The remaining solution was heated in a water bath. After evaporation, the samples were dried in the oven to constant weight and the saponin content was calculated [22].

#### 2.6.3. Total Phenolic Compounds Estimation

The content of total phenolic compounds of the extract was determined according to McDonald's method using Folin–Ciocalteau reagent (Gallic acid as a standard) [23].

#### 2.6.4. Dose- and Time-Dependent Effect of AEPD

To find out the dose of AEPD necessary for optimum protection against CCl_4_-induced hepato-toxicity mice were divided into 10 groups each consisting of six animals in each. First two groups were served as normal control (received only water as vehicle) and toxin control (received CCl_4_ at a dose of 1 ml kg^−1^ body weight for 2 days, orally), respectively. Other eight groups of animals were treated with AEPD orally at a dose of 25, 50, 75, 100, 150, 200, 250 and 300 mg kg^−1^ body weight for 7 days prior to CCl_4_ treatment (at a dose of 1 ml kg^−1^ body weight for 2 days, orally) respectively.

To determine the time dependent effects of AEPD against CCl_4_-intoxicated hepatic disorders, mice were divided into nine groups each consisting of six animals. First two groups were served as normal control (received only water as vehicle) and toxin control (received CCl_4_ at a dose of 1 ml kg^−1^ body weight for 2 days, orally) respectively. Other seven groups of animals were treated with AEPD orally at a dose of 200 mg kg^−1^ body weight, once daily for 1, 3, 5, 7, 10, 12 and 14 days prior to CCl_4_ intoxication (at a dose of 1 ml kg^−1^ body weight for 2 days, orally).

All mice were sacrificed 24 h after the final dose of CCl_4_ administration. The ALT levels were measured from the blood serum of all the experimental mice.

### 2.7. Experimental Animals Grouping and Treatment

Figure 1 represents the animals grouping and their treatment procedure. 

### 2.8. Liver Weight to Body Weight Ratio Determination

After scarification, the livers from experimental animals were quickly excised and weighed. The ratio of liver weight to body weight was then measured for each.

### 2.9. Serum Marker Enzymes Inhibition Efficiency

For the assessment of serum-specific markers (ALT and ALP) related to hepatic dysfunction, blood samples were collected by puncturing mice hearts of all experimental animals, kept overnight for clotting and then centrifuged at 3000 g for 10 min. ALT and ALP levels (in the sera) were measured by using the kits from Span Diagnostic limited, India.

### 2.10. Liver Tissue Homogenate Preparation

About 200 mg liver tissue was homogenized using glass homogenizer in 100 mM phosphate buffer (pH 7.4), containing 1 mM EDTA, PMSF (proteinase inhibitor, 1 mM) as well as phosphatase inhibitor cocktail (1 : 100 dilution) and the mixture was centrifugation at 12 000 g for 30 min at 4°C. The supernatant was collected and used for the experiments.

### 2.11. Tissue Homogenate Protein Content Determination

The protein contents of the liver tissue homogenates were measured by the method of Bradford using crystalline BSA as standard [24].

### 2.12. Lipid Peroxidation, Lipid Hydroperoxide and PC Inhibition Efficiency

The level of lipid peroxidation was measured in terms of the formation of thiobarbituric acid reactive substances (TBARS) according to the method of Esterbauer and Cheeseman [25]. Liver tissue homogenate, containing 1 mg protein, were mixed with 1 ml TCA (20%), 2 ml TBA (0.67%) and heated for 1 h at 100°C. During heating step 0.01% butylated hydroxyl toluene was added to abolish the metal catalyzes auto-oxidation of lipids. After cooling, the precipitate was removed by centrifugation. The pink pigment from all the samples was separately extracted with 4 ml of *n*-butanol. The absorbance of the sample was measured at 535 nm using a blank containing all the reagents except the sample. As 99% TBARS are malondialdehyde (MDA), so TBARS concentrations of the samples were calculated using the extinction co-efficient of MDA, which is 1.56 × 10^5^ M^−1^cm^−1^ [25].

The concentration of lipid hydroperoxide (LHP) in the experimental sample was estimated by the FOX reagent as described by Jiang et al. [26]. For this purpose, the tissue homogenate was mixed with FOX reagent [88 mg of butylated hydroxy toluene, 7.6 mg xylenol orange and 9.8 mg of ammonium iron (II) sulfate in 90 ml methanol and 10 ml of H_2_SO_4_]. After 30 min the absorbance of the solution was read at 560 nm. The amount of hydroperoxide produced was calculated using the molar extinction coefficient of 4.6 × 10^4^ M^−1^cm^−1^.

Protein carbonyl contents in the liver tissue samples were determined according to the method of Uchida and Stadtman [27]. The tissue homogenate was mixed with an equal volume of 0.1% (w/v) 2,4-DNPH in 2N HCl and incubated for 1 h at room temperature and then treated with 20% TCA. After centrifugation, the precipitate was extracted three times with ethanol/ethyl acetate and dissolved in 8 M guanidine hydrochloride in 133 mM Tris buffer containing 13 mM EDTA. The absorbance was recorded at 365 nm. The results were expressed as nanomoles of DNPH incorporated/mg protein based on the molar extinction coefficient of 22 000 M^−1^cm^−1^ for aliphatic hydrazones.

### 2.13. Antioxidant Enzymes and Metabolites Assay

#### 2.13.1. SOD

In case of SOD assay tissue homogenates were centrifuged at 600 g for 8 min at 4°C. Supernatants were decanted and re-centrifuged at 5500 g for 15 min to form mitochondrial pellets. The supernatant was kept as “cytosolic fraction". The pellets were resuspended in MSH buffer (210 mM mannitol, 70 mM sucrose, 5 mM Hepes, pH 7.5) without EDTA and termed as “mitochondrial fraction". The activities of Mn–SOD were measured in the mitochondrial and Cu/Zn–SOD in the cytosolic fractions following the method of Nishikimi et al. [28] and Kakkar et al. [29]. The addition of cyanide ion (in mitochondrial fraction) to a final concentration of 2 mM inhibits Cu/Zn–SOD activity by over 90%. Mn–SOD is unaffected by cyanide. For both measurements, about 5 *μ*g of protein was mixed with sodium pyrophosphate buffer, PMT and NBT. The reaction was started by the addition of NADH. The reaction mixture was then incubated at 30°C for 90 s and stopped by the addition of 1 ml of glacial acetic acid. The absorbance of the chromogen formed was measured at 560 nm. One unit of SOD activity is defined as the enzyme concentration required to inhibit chromogen production by 50% in 1 min under the assay condition.

#### 2.13.2. CAT

The enzyme CAT converts H_2_O_2_ formed via the action of SOD on superoxide radical into water. The CAT activity was measured by the method of Bonaventura et al. [30]. About 5 *μ*g protein from spleen homogenate was mixed with 2.1 ml of 7.5 mM H_2_O_2_ and a time scan was performed at 240 nm spectrophotometrically for 10 min at 25°C. The disappearance of peroxide depending on the CAT activity was observed. One unit of CAT activity is defined as the amount of enzyme, which reduces 1 *μ*mol of H_2_O_2_ per minute.

#### 2.13.3. GST

The activity of GST was measured by the method of Habig et al. [31]. The reaction mixture contained suitable amount of enzyme (25 *μ*g of protein in homogenates), potassium phosphate buffer, EDTA, CDNB and GSH. The reaction was carried out at 37°C and monitored spectrophotometrically by the increase in absorbance of the conjugate of GSH and CDNB at 340 nm. A blank was run in absence of the enzyme. One unit of GST activity is defined as the 1 *μ*mol of product formation per minute.

#### 2.13.4. GR

GR activity was determined according to the method of Smith et al. [32]. The increase in absorbance at 412 nm was monitored spectrophotometrically for 3 min at 24°C. The enzyme activity was calculated using molar extinction coefficient of 13 600 M^−1^cm^−1^. One unit of enzyme activity is defined as the amount of enzyme, which catalyzes the oxidation of 1 *μ*mol NADPH per minute.

#### 2.13.5. GPx

GPx activity was assayed according to the method of Flohe and Gunzler [33]. About 50 *μ*l of sample was mixed with 550 *μ*l of 0.1 M KH_2_PO_4_ buffer containing 1 mM EDTA (pH 7.5), 50 *μ*l of 2 mM NaN_3_, 100 *μ*l of GR (2.4 U ml^−1^) and 100 *μ*l of 10 mM GSH. After 10 min of incubation at 37°C, 100 *μ*l of 1.5 mM NADPH in water was added to the above mixture. The reaction was started by adding 100 *μ*l of pre-warmed (37°C) 1.5 mM H_2_O_2_ and the decrease in absorbance at 340 nm were monitored spectrophotometrically for 5 min. The enzyme activity was calculated using molar extinction coefficient of 6.22 × 10^3^ M ^−1^cm^−1^. One unit of enzyme activity is defined as the amount of enzyme that catalyzes the oxidation of 1 *μ* mol NADPH per minute.

#### 2.13.6. GSH

GSH level was measured by the method of Ellman [34]. Liver tissue homogenate (720 *μ*l) was diluted to 1440 *μ*l by using Tris-EDTA buffer and 5% TCA was added to it to precipitate the protein content of the homogenate. After centrifugation (10 000 g for 5 min) the supernatant was taken, DTNB solution (Ellman's reagent) was added to it and the absorbance was measured at 417 nm. A standard graph was drawn using different concentrations of GSH solution (1 mg ml^−1^) and fixed concentration of DTNB. With the help of this graph GSH content of tissue homogenates were calculated. The method describes here basically determines the total non-protein sulfhydryls (NPSH) in the experimental samples as proteins are precipitated initially by TCA. However, GSH is the most abundant NPSH in the tissue. Thus, the aforementioned method can be regarded as the GSH estimation procedure.

#### 2.13.7. GSSG

Glutathione disulfide (GSSG) was assessed by measuring its level using a kit from Calbiochem, USA following the method of Finck et al. [35]. In this method, GSSG was enzymatically reduced to GSH (in presence of NADPH and GR as given below) which reacts with DTNB to produce the yellow colored TNB

(1) $$\begin{array}{c} \text{GSSG}+\text{NADPH}+{\text{H}}^{+}\overset{\text{GR}}{\to }2\text{GSH}+\text{NADP}\\ \text{GSH}+\text{DTNB}\to \text{TNB}\;\;\left(\text{Yellow}\;\text{color}\right) \end{array}$$

Briefly, tissue samples were homogenized in ice cold m-phosphoric acid (100 g l^−1^, Fluka). This treatment resulted in the precipitation of the proteins. After allowing the mixture to stand for 5 min at room temperature, homogenates were centrifuged (10 000 g; 10 min at 4°C). Supernatants were frozen at –80°C until further analysis. Prior to the estimation of GSSG, neutralization was achieved by adding 5 *μ*l of triethanolamine (4 mmol l^−1^, Sigma Chemicals) to a 100 *μ*l supernatant. For GSSG assay, the thiol scavenging reagent 1-methyl-2-vinylpyridinium trifluoromethanesulfonate (M2VP) was used to mask GSH very rapidly. An amount of 10 *μ*l of M2VP was added to 100 *μ*l of neutralized supernatant. Then 100 *μ*l of the recycling reagent, which contained NADPH (0.30 mM), DTNB (0.225 mM) and GR (1.6 U ml^−1^) in a 100 mM phosphate/1 mM EDTA buffer (pH 7.4), was added. The change of absorbance was monitored at 412 nm for 3 min with a spectrophotometer. Standards and test samples were run in triplicate for each assay and the measurements were repeated three times. The reaction rate and calibration curves were used to calculate concentrations of GSSG.

### 2.14. Total Thiols

Total thiols (total protein bound as well as non-protein bound sulfhydryl groups) content was measured according to the method of Sedlak and Lindsay [36] with some modifications. About 50 *μ*l of the tissue homogenate was mixed with 0.6 ml of Tris-EDTA buffer and 40 *μ*l of 10 mM DTNB in methanol. The final volume was made up to 1 ml by adding methanol. The reaction mixture was incubated at room temperature for 20 min and the absorbance was measured at 412 nm. The content of total thiols was calculated using molar extinction coefficient of 13 600 M^−1^ cm^−1^.

### 2.15. Intracellular ROS Production Inhibition

Intracellular ROS production was estimated by using 2,7-dichlorofluorescein diacetate (DCFDA) as a probe following the method of LeBel and Bondy [37] as modified by Kim et al. [38]. DCFDA diffuses through the cell membrane where it is enzymatically deacetylated by intracellular esterases to the more hydrophilic nonfluorescent reduced dye dichlorofluorescin. In the presence of reactive oxygen metabolites, nonfluorescent DCFH rapidly oxidized to highly fluorescent product DCF. For *in vivo* study, 100 *μ*l of tissue homogenates were incubated with the assay media (20 mM Tris–HCl, 130 mM KCl, 5 mM MgCl_2_, 20 mM NaH_2_PO_4_, 30 mM glucose and 5 *μ*M DCFDA) at 37°C for 15 min. The formation of DCF was measured at the excitation wavelength of 488 nm and emission wavelength of 610 nm for 10 min by using fluorescence spectrophotometer (HITACHI, Model No. F4500) equipped with a FITC filter. Representative images of the fluorescent cell were taken under fluroscence microscope.

### 2.16. Cytochrome P450 Activity Study

The reaction mixture contained 100 *μ*g liver microsomal protein in a 100-*μ*l reaction system containing 0.4 mM *p*-nitrophenol and 1 mM NADPH. The reaction was incubated at 37°C and stopped after 60 min by addition of 30 ml 20% TCA and placed on ice. Briefly after centrifugation, the sup was taken and mixed with 2 M NaOH and the absorbance measured at 546 nm. 4-Nitrocatechol formation was quantitated by using an extinction coefficient of 10.28 mM^−1^ cm^−1^ [39].

### 2.17. Immunoblotting

Samples containing 50 *μ*g proteins were subjected to 10% SDS–PAGE and transferred to a nitrocellulose membrane. Membranes were blocked at room temperature for 2 h in blocking buffer containing 5% non-fat dry milk to prevent non-specific binding and then incubated with primary antibody, CYP2E1 (1 : 1000 dilution), overnight at 4°C. The membrane was washed in TBST (50 mmol l^−1^ Tris–HCl, pH 7.6, 150 mmol l^−1^ NaCl, 0.1% Tween 20) for 30 min and incubated with appropriate HRP conjugated secondary antibody (1 : 2000 dilution) for 2 h at room temperature and developed by the HRP substrate 3,3′-diaminobenzidine tetrahydrochloride (DAB) system (Bangalore, India).

### 2.18. DNA Damage Inhibition Analysis

The extent of DNA fragmentation (DNA ladder) has been assayed by electrophoresing genomic DNA samples, isolated from normal as well as experimental mouse liver, on agarose/ethydium bromide gel by the procedure described by Sellins and Cohen [40].

### 2.19. Detection of Cell Death Pathway by Flow Cytometry

The flow cytometric analysis was done on BD-LSR flow cytometer. Cell debris, characterized by a low FSC/SSC was excluded from analysis. The data was analyzed by Cell Quest software.

The apoptotic and necrotic cell distribution was analyzed by Annexin V binding and PI uptake. Positioning of quadrants on Annexin V/PI dot plots was performed and living cells (Annexin V^−^/PI^−^), early apoptotic/primary apoptotic cells (Annexin V^+^/PI^−^), late apoptotic/secondary apoptotic cells (Annexin V^+^/PI^+^) and necrotic cells (Annexin V^−^/PI^+^) were distinguished. Therefore, the total apoptotic proportion included the percentage of cells with fluorescence Annexin V^+^/PI^−^ and Annexin V^+^/PI^+^. The cells were suspended in 1 ml binding buffer (1x). An aliquot of 100 *μ*l was incubated with 5 *μ*l Annexin V-FITC and 10 l PI for 15 min in dark at room temperature and 400 *μ*l binding buffer (1x) was added to each sample. The FITC and PI fluorescence were measured through FL-1 filter (530 nm) and FL-2 filter (585 nm), respectively, and 10 000 events were acquired.

### 2.20. Histological Studies

Livers from the normal and experimental mice were fixed in 10% buffered formalin and were processed for paraffin sectioning. Sections of about 5 *μ*m thickness were stained with hematoxylin and eosin to evaluate under light microscope.

### 2.21. Free-Radical Scavenging Activity in Cell-Free System

#### 2.21.1. DPPH

The antioxidant activity of the aqueous extract was measured using the DPPH radical [41]. DPPH solutions (2 ml) in methanol (125 *μ*M) and 2 ml of tested samples with different concentrations were mixed in the tubes. The solution was shaken and incubated at 37°C for 30 min in dark. The decrease in absorbance at 517 nm was measured against methanol blank using a UV/Visible spectrophotometer. Percent inhibition was calculated by comparing the absorbance values of control and the sample. Percentage inhibition = ((*A*_1_ − *A*_2_)/*A*_2_) × 100, where *A*_1_ is the absorbance of the blank and *A*_2_ is the absorbance in the presence of the *P. Dulce* extract. A parallel experiment was carried out under the same conditions in which *P. Dulce* extract was replaced by vitamin C and used as a positive control.

#### 2.21.2. Hydroxyl

The hydroxyl radical scavenging activity of the extract has been investigated following the method of Nash [42]. *In vitro* hydroxyl radicals were generated by Fe^3+^/ascorbic acid system. The detection of hydroxyl radicals was carried out by measuring the amount of formaldehyde produced from the oxidation of dimethyl sulfoxide (DMSO). The formaldehyde produced was detected spectrophotometrically at 412 nm.

#### 2.21.3. Superoxide

The superoxide radical scavenging activity was measured following the method of Siddhuraju and Becker [43]. The reaction mixture contained 0.1 M phosphate buffer, pH 7.4, 150 *μ*M nitroblue tetrazolium (NBT), 60 *μ*M phenazine methosulphate (PMT), 468 *μ*M NADH and different concentrations of the AEPD. The mixture was incubated in the dark for 10 min at 25°C and the absorbance was read at 560 nm. Results were expressed as percentage inhibition of the superoxide radicals.

### 2.22. Statistical Analysis

All the values are expressed as mean ± SD (*n* = 6). Significant differences between the groups were determined with SPSS 10.0 software (SPSS Inc., Chicago, IL, USA) for Windows using one-way analysis of variance (ANOVA) and the group means were compared by Student-Newman-Keuls *post hoc* tests. A difference was considered significant at the *P* < .05 level.

## 3. Results

### 3.1. Phytochemical Screening of AEPD for Active Components

The present study investigated the presence of medicinally active constituents in the fruit extract. Qualitative analysis (Table 1) revealed that flavonoids, saponins, phenolics and steroids were present in the fruit extract of the plant. Quantitative estimation of the chemical constituents in the studied medicinal plant is summarized in Table 2. 

### 3.2. Dose- and Time-Dependent Protective Action of AEPD against CCl_4_ Intoxication

In the present study, we used ALT assay to determine the optimum dose and time necessary for AEPD to protect mouse liver against CCl_4_-induced hepatic oxidative damages. The experimental results of this study have been represented in Figures 2 and 3, respectively. Results show that CCl_4_ intoxication significantly increased the ALT activity in serum. AEPD administration decreased the ALT activity linearly up to a dose of 200 mg kg^−1^ body weight, when applied for 5 days prior to CCl_4_ intoxication. This dose of AEPD and time of treatment were used for the subsequent experiments. 

### 3.3. Liver Weight to Body Weight Ratio

CCl_4_ intoxication usually reduces the weight of different organs in pathophysiological situations. We, therefore, checked whether the liver weight of the experimental animals was affected by CCl_4_ exposure and if that happened whether AEPD could protect it.  Table 3 shows that CCl_4_ toxicity lowers liver weight to body weight ratio (*∼*30%) and that could be prevented by the treatment with AEPD prior to toxin exposure. Post-treatment with AEPD also showed similar result as the pre-treated groups. It is evident from the data that CCl_4_-induced hepatic pathophysiology could be protected by AEPD. 

### 3.4. Serum-Specific Markers Related to Hepatic Dysfunction

Table 3 represents the status of the serum specific marker enzymes related to liver dysfunction. CCl_4_ administration caused a significant increase in the activities of ALT (*∼*2-fold) and ALP (*∼*3-fold). Pre-treatment with AEPD could maintain these levels almost close to normal against CCl_4_-induced hepatotoxicity. Post treatment with AEPD after toxin administration also decreased these levels. Results suggest that AEPD could block the membrane leakage induced by CCl_4_-exposure.

### 3.5. Lipid Peroxidation and PC Inhibition

In oxidative-stress-related organ pathophysiology, lipid peroxidation and PC are considered to be the two important parameters. In the present study, lipid peroxidation has been measured by estimating the concentration of TBARS and LHP.  Table 4 represents the changes in TBARS, LHP and PC in the hepatic tissue of the normal and experimental animals. CCl_4_ intoxication increased the levels of TBARS (*∼*2.3-fold) and LHP (*∼*2-fold). The level of PC was also significantly elevated (*∼*2.4-fold) due to CCl_4_ toxicity. However, both pre- and post-treatment with AEPD decreased the levels of lipid peroxidation as well as PC suggesting the anti-oxidant nature of AEPD in CCl_4_-induced hepatic oxidative stress. 

### 3.6. Protective Role Against CCl_4_-Induced Intracellular ROS Production

ROS plays a major role in CCl_4_-induced hepatic dysfunction and hepatocellular death. In order to asses the changes in the production of intracellular ROS under oxidative stress, hepatocytes were isolated from the experimental animals and studied the ROS production assay using DCFDA under fluorescence microscope and by fluorescence spectrophotometer also.  Figure 4 shows the effect of CCl_4_ on the intracellular ROS production and its reversal by the treatment with AEPD. Here, we observed (Figure 4) that CCl_4_ administration caused increased production of intracellular ROS (*∼*80% as revealed by the increased no of green fluorescent cells). Treatment with AEPD both pre- and post-toxin administration decreased (*∼*40%) the intracellular ROS level compared to toxin control suggesting the intracellular ROS scavenging nature of AEPD. Data from fluorescence spectrophotometric analysis also supported this result. 

### 3.7. Antioxidant Enzymes Activation

Antioxidant enzymes are considered to be the first line of cellular defense that prevents cellular ingredients from oxidative damage. Among them SOD and CAT mutually function as important enzymes in the elimination of ROS. In order to remove excess free radicals from the system, GST and GPx utilize GSH during their course of reactions. Decrease in GSH content due to toxicity simultaneously decreased the activities of GST as well as GPx with a concomitant decrease in the activity of GSH regenerating enzyme, GR. We, therefore, determined the activities of these enzymes and presented the data in Table 5. A significant reduction in the activities of all antioxidant enzymes was observed in the liver tissue of the CCl_4_-intoxicated experimental animals. Results suggest that both pre- as well as post-treatment with AEPD could protect the first line of hepato-cellular defense in oxidative damage induced by CCl_4_. 

### 3.8. Cellular Metabolites Alterations

Thiol based antioxidant system plays second line of cellular defense against reactive free radicals and other oxidant species mediated oxidative damage. GSH with its –SH group functions as a catalyst in disulfide exchange reaction. It functions by scavenging free radicals as well as detoxifying various xenobiotics and consequently converted to its oxidized form, glutathione disulfide (GSSG). Levels of cellular metabolites like GSH, GSSG and total thiol have been described in Table 6. The levels of GSH and total thiols were significantly decreased (GSH *∼*71% and total thiols *∼*50%) due to CCl_4_ intoxication along with the increased (*∼*1.7-fold) level of GSSG. Pretreatment with AEPD could prevent the toxin-induced alterations in the intracellular thiol status. Post treatment with AEPD also maintained the levels of cellular metabolites close to normal suggesting the protective nature of AEPD for second line of hepato-cellular defense against free radicals and other oxidant species originated due to CCl_4_ exposure. 

A well-known antioxidant, vitamin C, has been included in the present study as a positive control. Being an antioxidant, vitamin C could prevent CCl_4_-induced hepatic oxidative dysfunction.

### 3.9. Upregulation of Cytochrome P450 and CYP2E1

The reactive metabolite trichloromethyl radical (^•^CCl_3_) has been formed from the metabolic conversion of CCl_4_ by cytochrome P450. As O_2_ tension rises, a greater fraction of ^•^CCl_3_ reacts very rapidly with O_2_ and more reactive free radical, CCl_3_OO^•^ has been generated from ^•^CCl_3_. CYP2E1, major isozyme of cytochrome P450 family, is involved in CCl_4_ bioactivation and generation of cytotoxic trichloromethyl radicals, caused hepatotoxicity [44–46]. Alterations in CYP2E1 activity can affect susceptibility to hepatic injury from CCl_4_ [46, 47]. Moreover, the reactive free radicals inactivate CYP enzymes and cause depletion of CYP2E1 [48–50].  Figure 4 shows the activity of cytochrome P450 and the expression of CYP2E1 in the liver tissue of different experimental animals. We observed (Figure 5) a reduced activity of cytochrome P450 (*∼*60%) as well as the expression of CYP2E1 (*∼*72%) (Figure 6) in the liver tissue of CCl_4_ intoxicated animals. Treatment with AEPD only has no effect on the activity of cytochrome P450 and the expression of CYP2E1 however when it is applied both pre- or post-toxin exposure then a significant increased the activity of cytochrome P450 and the expression of CYP2E1 was observed compared to the toxin group. This finding thus suggested the radical scavenging and antioxidant role of AEPD. 

### 3.10. DNA Damage Inhibition Efficiency

Oxidative stress induced by oxygen-derived species can produce a multiplicity of modifications in DNA including base and sugar lesions, strand breaks, DNA-protein cross-links and base-free sites. If left un-repaired, oxidative DNA damage can lead to detrimental biological consequences in organisms, including cell death, mutations and transformation of cells to malignant cells. In order to find out whether AEPD protects CCl_4_-induced DNA damage, DNA fragmentation was examined by agarose gel electrophoresis.  Figure 7 represents the results. A smear on agarose gel had been observed in CCl_4_-treated group, indicating random DNA fragmentation, a hallmark of necrosis. AEPD pretreatment found to be effective to prevent the toxin-induced smear formation suggesting that AEPD possesses the protective power for the prevention of liver cells from CCl_4_-induced DNA damage and necrotic death. 

### 3.11. Cell Death Pathways

To understand the nature of cell death due to CCl_4_ toxicity, double labeling techniques has been utilized using Annexin V/PI to distinguish between apoptotic and necrotic cells. Flowcytometric data (Figure 8) revealed that, in comparison with control untreated hepatocytes, hepatocytes isolated from CCl_4_-intoxicated mice showed maximum PI staining (*∼*55%), but very little Annexin V-FITC-binding (*∼*5%) indicating majority of cell death occurs via necrotic pathway. In AEPD pretreated group the number of necrotic cells was significantly low indicating the extract pre-treatment prevented the hepatocytes from CCl_4_-induced necrotic cell death. Post-treatment with AEPD also reduced the CCl_4_-induced cell death via necrotic pathway.

### 3.12. Histological Assessment

Histological assessments of different liver segments of the normal and experimental animals have been presented in Figure 9. CCl_4_ exposure induced necrosis along the central vein and disorganized the normal radiating pattern of cell plates around it. Treatment with AEPD prior to and after the toxin exposure showed a considerable improvement in liver morphology. Results of the histological assessment support the outcome of the earlier studies by exhibiting CCl_4_-induced necrosis in the liver tissue and its protection by AEPD. 

### 3.13. Radical Scavenging Activity in Cell Free System

#### 3.13.1. DPPH

To begin with the evaluation of the antioxidant nature of AEPD, we looked for an effective radical scavenging cell free assay. So, we determined its radical scavenging power using the DPPH radical. The experimental results on the radical scavenging effect of AEPD have been shown in the Figure 10. The plot shows that with increase in concentration of AEPD the color of the DPPH radical vanishes rapidly at 517 nm. It has been observed that AEPD showed maximum inhibition when it was incubated at a concentration of 20 mg ml^−1^ with DPPH solution. Hence, it can be anticipated that the active principle(s) present in AEPD possesses potent free radical scavenging activity. 

#### 3.13.2. Hydroxyl (OH^•^) and Super oxide (O_2_^*•*^)

In addition to the DPPH radical scavenging activity, hydroxyl and superoxide radicals scavenging activity of AEPD has also been investigated in cell free system and Figure 11 represent those results. It has been observed that at a dose of 20 mg ml^−1^, AEPD can effectively scavenge OH^•^ and O_2_^*•*^ radicals. During the preparation of the plant extract, the extraction with phosphate buffer followed by lyophilization leave some superoxide dismutase which could be responsible for the superoxide radical scavenging activity of the extract. 

## 4. Discussion

In our body, liver is the major organ responsible for the metabolism of drugs and toxic chemicals and thus it is the primary target organ for nearly all toxic chemicals. Various pharmacological or chemical substances (such as acetaminophen, galactosamine, chloroform, dimethylnitrosamine, etc.) are known to cause hepatic injuries. Excessive exposure to these chemicals may cause acute liver injury characterized by abnormality of hepatic function, and degeneration, necrosis or apoptosis of hepatocytes, and so forth. In modern civilization drugs or chemicals induced liver injury has become a serious clinical problem. CCl_4_-induced liver injury in one of the well established system for xenobiotic-induced hepatotoxicity and is commonly used model for screening of the anti-hepatotoxic and/or hepatoprotective activities of the drugs. Present study investigated the protective role of AEPD against CCl_4_-induced hepatic disorders. It has been observed that CCl_4_ administration caused hepatic oxidative stress and cellular death mostly via the necrotic pathway. Treatment with AEPD both pre- and post-CCl_4_ administration prevented the toxin-induced hepatic damage.

Reduction in the liver weight to the body weight ratio and increased activities of the serum marker enzymes ALT, ALP are the two important physiological indices for hepatic injury. CCl_4_ administration caused reduction in the ratio of liver weight to body weight. However, both pre- and post-treatment with AEPD were effective to keep the ratio of the liver weight to the body weight almost close to normal. Membrane permeability is altered due to the hepatocytes injury, leading to leakage of enzymes from these cells during toxin and drug-induced hepatotoxicity. Hepatocellular damage, as evident from a significant elevation in serum activities of ALT and ALP, used as reliable markers of hepatotoxicity. In our study CCl_4_ intoxication increased the levels of serum marker enzymes (ALT and ALP) indicating the severity of hepatocellular damage induced by CCl_4_. Treatment with AEPD in this intoxication reduced the activities of ALT as well as ALP and thus maintained the integrity of the cellular membrane close to normal.

Increased production of intracellular ROS plays a major role in CCl_4_-induced hepato-cellular damage. We observed that CCl_4_ exposure increased the production of intracellular ROS as evidenced by the increased number of green fluorescent cells. Increased level of ROS induced by CCl_4_ suggested a higher degree of oxidative stress and extent of cellular damage in hepatic tissues. Treatment with AEPD against CCl_4_ exposure reduced the increased production of intracellular ROS and thus kept the liver tissue normal in normal physiology.

Over production of ROS initiates the process of lipid peroxidation in cell membranes and cause destruction of cell components as well as cell death [51]. Lipid peroxidation and PC are considered to be the two important parameters of oxidative stress. Lipid peroxidation was measured by estimating the concentrations of TBARS as well as LHP. Several reports have shown that hepatic lipid peroxidation increases with the development of acute liver injury in rats treated once with CCl_4_ [52, 53]. In our study we found that CCl_4_ intoxication increased the levels of TBARS, LHP and PC in the hepatic tissue of the experimental animals. Treatment with AEPD both pre- and post-CCl_4_ administration attenuated the increased levels of the lipid peroxidation and PC.

The intracellular defense mechanism comprises of various antioxidant enzymes (SOD, CAT along with GSH dependent enzymes, GST, GR and GPx). The antioxidant enzyme, SOD quenches O_2_^−^ by converting it into O_2_ and H_2_O_2_ and CAT converts H_2_O_2_ into H_2_O and O_2_. GST helps in the radical scavenging reaction of GSH. GR catalyses the conversion of GSH from GSSG and GPx helps to consume of H_2_O_2_ by reaction with GSH. Therefore, in order to eliminate the free radicals, these cellular antioxidant enzymes play an important role and equilibrium exists between these enzymes under normal physiological conditions. CCl_4_ exposure decreased the activities of all the antioxidant enzymes. AEPD treatment against CCl_4_ administration significantly restored the altered activities of all antioxidant enzymes.

GSH, considered as the second line of intracellular defense system with its sulfhydryl group (–SH) is a catalyst in disulfide exchange reaction. It scavenges free radicals and ROS as well as detoxifies various xenobiotics and consequently converted itself to its oxidized form, glutathione disulfide (GSSG). Thus, reduction of GSH is associated with a rise in GSSG concentration resulting with the depletion in GSH/GSSG ratio. In the present study, we observed that CCl_4_ intoxication decreased the levels of GSH and simultaneously increased the level of GSSG suggesting a clear role of oxidative stress in CCl_4_-induced hepatic pathophysiology. However, both pre- and post-treatment with AEPD normalized all the levels as compared to the respective controls.

It has been established that CCl_4_-induced hepatotoxicity depends on its reductive dehalogenation, catalyzed by the cytochrome P450 enzymes, in the endoplasmic reticulum of hepatic cells, leading to the generation of an unstable complex trichloromethyl radical. The trichloromethyl radical may bind either at the heme group of cytochrome P450 or at the active site of the enzyme near the heme group, leading to the inactivation P450 pathways [54]. Among the different cytochrome P450 enzymes CYP2E1 play a major role in the bioactivation of CCl_4_. CYP2E1-mediated metabolism of CCl_4_ generated reactive free radicals and CYP2E1 protein might be more susceptible to CCl_4_ toxicity than other CYP isozymes. In the present study a significant decreased activity of cytochrome P450 and the expression of CYP2E1 were found in the hepatic tissues of CCl_4_ intoxicated animals, suggesting that CYP2E1 was degraded during the process of CCl_4_-induced hepatotoxicity. Treatment with AEPD however prevented the degradation of cytochrome P450 and CYP2E1 as well as bioactivation of CCl_4_ and thus protected the liver tissue against CCl_4_-induced hepatic damage.

DNA strand breaks can originate from the direct modification of DNA by chemical agents or their metabolites; from the processes of DNA excision repair, replication and recombination; or from the process of apoptosis [55]. Direct breakage of the DNA strands occurs when reactive oxygen species interact with DNA [56]. The mode of cell death induced by CCl_4_ was investigated using DNA fragmentation as well as flow cytometric analyses and checked whether AEPD treatment would reduce it or not. In our study we found that CCl_4_ exposure induced random fragmentation of genomic DNA, causing formation of a DNA smear on agarose gel. In addition to the DNA fragmentation study, flow cytometric analysis showed that CCl_4_ exposure increased the population of PI staining cells compared to the annexin-V staining cells. Thus both the smear on agarose gel and increased number of PI staining cell indicate the CCl_4_-induced cell death via necrotic pathway. Treatment with AEPD, however, decreased the degree of CCl_4_-induced necrotic cell death and protected the liver from the adverse effect of the toxin.

Although the liver is the principal site for CCl_4_-induced toxicity, but there is no specific “receptor" for the actions of CCl_4_. Pathological changes following CCl_4_ poisoning have been identified at the biochemical and the ultra structural level [57, 58].

Histological studies showed that CCl_4_-intoxication caused considerable necrosis in the liver tissue along the central vein. The necrosis was mostly centrilobular and extending through the whole liver lobule. AEPD administration both pre- and post-CCl_4_ intoxication reduced the toxin-induced centrilobuler necrosis and thus protected the organ.

DPPH radical scavenging assay is a convenient tool for the determination of free radical scavenging property of a compound in cell free system [41]. Incubation of AEPD at various concentrations with DPPH radical diminished the absorbance at 517 nm. This experiment reveals the ability of AEPD to scavenge DPPH radicals. In addition, we also investigated the hydroxyl as well as superoxide radicals scavenging activity of AEPD in cell-free system. Results of these studies clearly showed the free-radical scavenging activity of AEPD. It is therefore possible that in CCl_4_-induced hepato-cellular damage, AEPD acts as a free-radical scavenger which alters toxic effects of CCl_4_ by quenching the excessive free radicals.

It has been reported [59] that the fruits of *P. dulce* contain about 2.5% protein, 0.4% fat, 18% carbohydrate, 77.8% water and 1.3% fiber. Besides, *∼*77.8 calories can be obtained from 100 g fruits of *P. dulce*. It also contains some essential minerals like Ca, P, Fe, Na and K. It is also enriched with vital vitamins like thiamine, riboflavin, niacin and ascorbic acid. Few essential amino acids like valine, lysine, phenylalanine and tryptophan have also been found in this fruit. Alcoholic extraction yielded saponin, sterol glucoside, flavone and lecithin. In our study we also verified the presence of flavonoids, saponins, phenolics and steroids in the plant extract. The observed effects of the plant extract could be related to chemically defined compounds. Flavonoids show their antioxidative action through scavenging or chelating process. Phenolic content is also very important plant constituent because of their scavenging ability due to their hydroxyl groups. Thus the observed antioxidant effects could be related to the presence of flavonoid and phenolic content of the extract.

Figure 12 shows the possible mechanistic pathways about the beneficial role of AEPD against CCl_4_-induced hepatic pathophysiology. Here it has been observed that free radical scavenging activity of AEPD prevented the toxin induced over production of ROS. Besides, inhibition of the degradation of cytochrome P450 isoenzymes also reduced the bioactivation of CCl_4_ and its metabolite. Thus AEPD plays a protective role against CCl_4_-induced hepatic impairment via reducing oxidative stress and degradation of cytochrome P450s. 

In conclusion, we would like to mention that AEPD could be a useful agent against CCl_4_-induced hepatic pathophysiology (Figure 12). However, further studies are necessary to entirely characterize the active ingredient(s) of this fruit as well as the exact mechanism(s) of its protective action.

## Figures and Tables

**Figure 1:** Schematic diagram of in vivo experimental protocol. CCl_4_ was administered orally at a dose of 1 ml kg^−1^ body weight in liquid paraffin (1 : 1, v/v). AEPD and vitamin C were administered at a dose of 200 and 100 mg kg^−1^ body weight, respectively. The animals were sacrificed under light ether anesthesia at the specified time as mentioned in the figure.

**Figure 2:** Dose dependent effect of AEPD on ALT activity against CCl_4_-induced hepato-toxicity. Vehicle: ALT activity in normal mice, CCl_4_: ALT activity in CCl_4_-treated mice, AEPD-25, AEPD-50, AEPD-75, AEPD-100, AEPD-150, AEPD-200, AEPD-250, AEPD-300: ALT activity in AEPD-treated mice for 7 days at a dose of 25, 50, 75, 100, 150, 200, 250 and 300 mg kg^−1^ body weight prior to CCl_4_ intoxication. Data are mean ± SD, for six animals per group and were analyzed by one-way ANOVA, with Student-Newman-Keuls *post hoc* tests. Differences were attributed at *P* < .05, and homogeneous subgroups share common superscripted letters.

**Figure 3:** Time dependent effect of AEPD on ALT activity against CCl_4_-induced hepato-toxicity. Vehicle: ALT activity in normal mice, CCl_4_: ALT activity in CCl_4_-treated mice, AEPD-1, AEPD-3, AEPD-5, AEPD-7, AEPD-10, AEPD-12 and AEPD-14: ALT activity in AEPD-treated mice at a dose of 200 mg kg^−1^ body weight prior to CCl_4_ intoxication for 1, 3, 5, 7, 10, 12 and 14 days respectively. Data are mean ± SD, for six animals per group and were analyzed by one-way ANOVA, with Student-Newman-Keuls *post hoc* tests. Differences were attributed at *P* < .05, and homogeneous subgroups share common superscripted letters.

**Figure 4:** The intracellular ROS production was detected by DCF-DA method. (a) Representative images under fluroscence microscope (original magnification 400x), (b) intensity of DCF fluorescence (indicator of intracellular ROS level) measured using a fluorescence spectrophotometer. Vehicle: ROS level in normal animals, AEPD: ROS level in the animals treated with AEPD only; CCl_4_: ROS level in the CCl_4_ intoxicated animals; AEPD + CCl_4_: ROS level in the animals treated with AEPD prior to CCl_4_ intoxication; CCl_4_ + AEPD: ROS level in the animals treated with AEPD post-CCl_4_ intoxication and Recovery: ROS level in the animals of recovery group. Data are mean ± SD, for six animals per group and were analyzed by one-way ANOVA, with Student-Newman-Keuls *post hoc* tests. Differences were attributed at *P* < .05, and homogeneous subgroups share common superscripted letters.

**Figure 5:** Effect on the activities of cytochrome P450 in the hepatic tissue of the experimental animals. Vehicle: activity in normal animals, AEPD: activity in the animals treated with AEPD only; CCl_4_: activity in the CCl_4_ intoxicated animals; AEPD + CCl_4_: activity in the animals treated with AEPD prior to CCl_4_ intoxication; CCl_4_ + AEPD: activity in the animals treated with AEPD post-CCl_4_ intoxication and Recovery: activity in the animals of recovery group. Data are mean ± SD, for six animals per group and were analyzed by one-way ANOVA, with Student-Newman-Keuls *post hoc* tests. Differences were attributed at *P* < .05, and homogeneous subgroups share common superscripted letters.

**Figure 6:** Western blot analysis of the expression of CYP2E1 in the hepatic tissue of the experimental animals. The relative bands intensities were determined using NIH image software and the control band was given an arbitrary value of 1. Vehicle: CYP2E1 expression in normal animals, AEPD: CYP2E1 expression in the animals treated with AEPD only; CCl_4_: CYP2E1 expression in the CCl_4_ intoxicated animals; AEPD + CCl_4_: CYP2E1 expression in the animals treated with AEPD prior to CCl_4_ intoxication; CCl_4_ + AEPD: CYP2E1 expression in the animals treated with AEPD post-CCl_4_ intoxication and Recovery: CYP2E1 expression in the animals of recovery group. Data are mean ± SD, for six animals per group and were analyzed by one-way ANOVA, with Student-Newman-Keuls *post hoc* tests. Differences were attributed at *P* < .05, and homogeneous subgroups share common superscripted letters.

**Figure 7:** DNA fragmentation on agarose/ethydium bromide gel. DNA isolated from experimental liver tissues was loaded onto 1% (w/v) agarose gels. Lane 1: Marker (1-kb DNA ladder); lane 2: DNA isolated from vehicle; lane 3: DNA isolated from AEPD-treated liver samples; lane 4: DNA isolated from CCl_4_ intoxicated liver; lane 5: DNA isolated from AEPD pretreated liver samples; lane 6: DNA isolated from liver sample of the AEPD post-treated mouse and lane 7: DNA isolated from liver sample of the mouse of recovery group.

**Figure 8:** Representative flow cytometric analysis of hepatocytes from experimental animals. Vehicle: hepatocytes from normal animals, AEPD: hepatocytes from the animals treated with AEPD only; CCl_4_: hepatocytes from the CCl_4_ intoxicated animals; AEPD + CCl_4_: hepatocytes from the animals treated with AEPD prior to CCl_4_ intoxication; CCl_4_ + AEPD: hepatocytes from the animals treated with AEPD post-CCl_4_ intoxication, Recovery: hepatocytes from the animals of recovery group and NaAsO_2_: hepatocytes from the NaAsO_2_ intoxicated (100 ppm in drinking water, 10 weeks) animals (Positive control). Dual parameter dot plot of FITC-lebelled Annexin V fluorescence (*x*-axis) versus PI-fluorescence (*y*-axis) has been shown in logarithmic fluorescence intensity. Quadrants: lower left, live cells; lower right, apoptotic cells; upper left, necrotic cells. Data are representative of three independent experiments.

**Figure 9:** Hematoxylin and eosin stained liver section of experimental mice. (Cont) liver section from vehicle mice (100x); (AEPD) liver section of the mice treated with AEPD only (100x); (CCl_4_) mice administered with CCl_4_ (100x) (arrows indicate centrilobuler necrosis extending throughout the lobule associated with severe cellular damage); (AEPD + CCl_4_) liver section from the AEPD pre-treated mice (100x); (CCl_4_ + AEPD) liver section from the AEPD post-treated mice (100x) and (recovery) liver section from the mice of recovery group (100x).

**Figure 10:** DPPH radical scavenging activity of AEPD in cell free system. Each measurement was made six times. Data represent the average ± SD of six separate experiments. Asterisk indicates the optimum dose of AEPD at which it shows its maximum DPPH radical scavenging activity.

**Figure 11:** Hydroxyl (black square) and superoxide radical (red circle) scavenging activities of AEPD in cell free system. Each measurement was made six times. Data represent the average ± SD of six separate experiments. Asterisk indicates the optimum dose of AEPD at which it shows its maximum hydroxyl and superoxide radicals scavenging activities.

**Figure 12:** Schematic diagram of the antioxidative role AEPD and its protective role against CCl_4_-induced hepatic pathophysiology.

**Table 1:** Qualitative analysis of the AEPD.

Serial No.	Component	Abundance
1	Flavonoids	+
2	Saponins	+
3	Phenolics	+
4	Steroids	+

“+" sign indicates the presence of the compounds in the AEPD.

**Table 2:** Quantitative analysis of the AEPD.

Serial No.	Component	Concentration
1	Flavonoid content	55.47 ± 1.57
	(mg g^−1^ dry weight material)	
2	Saponin content	72.81 ± 2.35
	(mg g^−1^ dry weight material)	
3	Phenol content	3.12 ± 0.08
	(mg ml^−1^)	

**Table 3:** Ratio of the liver weight to the body weight and the activities of the serum marker enzymes related to hepatic dysfunction.

Animal groups	Ratio of the liver weight to the body weight (%)	Activities of the serum marker enzymes	
		ALT	ALP
Vehicle	4.78 ± 0.26^(a)^	46.22 ± 2.42^(a)^	25.88 ± 1.32^(a)^
AEPD	4.72 ± 0.25^(a)^	49.15 ± 2.47^(a)^	28.95 ± 1.28^(a)^
CCl_4_	3.33 ± 0.18^(b)^	97.39 ± 4.88^(b)^	75.77 ± 3.82^(b)^
AEPD + CCl_4_	4.45 ± 0.24^(a)^	54.58 ± 2.75^(a)^	52.98 ± 2.66^(c)^
CCl_4_ + AEPD	4.29 ± 0.26^(a)^	62.37 ± 3.12^(a)^	55.29 ± 2.77^(c)^
VitC + CCl_4_	4.55 ± 0.29^(a)^	50.49 ± 2.55^(a)^	44.15 ± 2.22^(c)^
Recovery	3.65 ± 0.17^(b)^	87.31 ± 4.39^(b)^	70.56 ± 3.55^(b)^

ALT: IU l^−1^ and ALP: KA. Data are mean ± SD, for six animals per group and were analyzed by one-way ANOVA, with Student-Newman-Keuls *post hoc* tests. Differences were attributed at *P* < .05, and homogeneous subgroups share common superscripted letters.

**Table 4:** Levels of the parameters as the index of lipid peroxidation (TBARS), LHP and PC in the liver tissue of the control and experimental mice.

Animal groups	TBARS	LHP	PC
Vehicle	7.37 ± 0.39^(a)^	2.35 ± 0.14^(a)^	18.91 ± 0.98^(a)^
AEPD	8.14 ± 0.42^(a)^	2.41 ± 0.12^(a)^	18.45 ± 0.95^(a)^
CCl_4_	17.25 ± 0.91^(b)^	4.76 ± 0.25^(b)^	45.51 ± 2.31^(b)^
AEPD + CCl_4_	9.14 ± 0.47^(a),(c)^	3.55 ± 0.19^(c)^	20.14 ± 1.03^(a)^
CCl_4_ + AEPD	10.37 ± 0.55^(c)^	3.12 ± 0.17^(a)^	25.95 ± 1.05^(a)^
VitC + CCl_4_	8.75 ± 0.45^(a)^	2.89 ± 0.15^(a)^	19.75 ± 0.98^(a)^
Recovery	15.29 ± 0.77^(b)^	4.51 ± 0.22^(b)^	42.25 ± 2.29^(b)^

TBARS—nmol mg^−1^ protein; LHP—nmol mg^−1^ protein and PC—nmol mg^−1^ protein. Data are mean ± SD, for six animals per group and were analyzed by one-way ANOVA, with Student-Newman-Keuls *post hoc* tests. Differences were attributed at *P* < .05, and homogeneous subgroups share common superscripted letters.

**Table 5:** Effect of CCl_4_ and AEPD on the activities of the antioxidant enzymes in liver tissue of the normal and experimental animals.

Animal Groups	Cu/Zn SOD	Mn SOD	CAT	GST	GR	GPx
Vehicle	75.12 ± 3.65^(a)^	65.73 ± 3.33^(a)^	47.05 ± 2.35^(a)^	2.25 ± 0.21^(a)^	11.17 ± 0.55^(a)^	91.47 ± 4.62^(a)^
AEPD	69.67 ± 3.41^(a)^	59.25 ± 3.01^(a)^	40.57 ± 2.02^(a)^	2.12 ± 0.17^(a)^	10.23 ± 0.41^(a)^	87.39 ± 4.44^(a)^
CCl_4_	26.54 ± 2.04^(b)^	16.38 ± 0.95^(b)^	15.27 ± 0.76^(b)^	0.85 ± 0.09^(b)^	3.18 ± 0.23^(b)^	44.25 ± 2.25^(b)^
AEPD + CCl_4_	54.62 ± 2.81^(a),(c)^	50.12 ± 2.55^(a),(c)^	35.23 ± 1.76^(a),(c)^	1.95 ± 0.15^(a)^	9.41 ± 0.47^(a)^	81.21 ± 4.12^(a)^
CCl_4_ + AEPD	49.75 ± 2.51^(c)^	45.56 ± 2.31^(c)^	31.55 ± 1.62^(c)^	1.75 ± 0.12^(a)^	8.75 ± 0.49^(a)^	76.91 ± 3.87^(a)^
VitC + CCl_4_	60.35 ± 3.05^(a)^	55.17 ± 2.78^(a)^	38.39 ± 1.92^(a)^	2.05 ± 0.14^(a)^	10.51 ± 0.53^(a)^	85.73 ± 4.33^(a)^
Recovery	30.12 ± 1.52^(b)^	20.43 ± 1.04^(b)^	18.35 ± 0.95^(b)^	0.91 ± 0.11^(b)^	3.22 ± 0.18^(b)^	48.31 ± 2.45^(b)^

SOD—U mg^−1^ protein; CAT—*μ*mol min^−1^ mg^−1^ protein; GST—*μ*mol min^−1^ mg^−1^ protein; GR–nmol min^−1^ mg^−1^ protein and GPx—nmol min^−1^ mg^−1^ protein. Data are mean ± SD, for six animals per group and were analyzed by one-way ANOVA, with Student-Newman-Keuls *post hoc* tests. Differences were attributed at *P* < .05, and homogeneous subgroups share common superscripted letters.

**Table 6:** Status of the thiol-based antioxidant in the liver tissue of the CCl_4_- and AEPD-treated animals.

Animal groups	GSH	GSSG	Total thiols
Vehicle	29.53 ± 1.52^(a)^	3.45 ± 0.19^(a)^	315.31 ± 15.76^(a)^
AEPD	25.74 ± 1.29^(a)^	3.51 ± 0.18^(a)^	305.25 ± 15.31^(a)^
CCl_4_	8.34 ± 0.45^(b)^	5.75 ± 0.28^(b)^	155.89 ± 7.85^(b)^
AEPD + CCl_4_	21.45 ± 1.09^(a),(c)^	3.85 ± 0.19^(a)^	255.34 ± 12.74^(a)^
CCl_4_ + AEPD	18.74 ± 0.95^(c)^	4.01 ± 0.21^(a)^	275.55 ± 13.79^(a)^
VitC + CCl_4_	23.45 ± 1.21^(a)^	3.69 ± 0.18^(a)^	297.31 ± 14.92^(a)^
Recovery	9.15 ± 0.49^(b)^	5.55 ± 0.27^(b)^	168.52 ± 8.45^(b)^

GSH—nmol mg^−1^ protein; GSSG—nmol mg^−1^ protein and total thiols—nmol mg^−1^ protein. Data are mean ± SD, for six animals per group and were analyzed by one-way ANOVA, with Student-Newman-Keuls *post hoc* tests. Differences were attributed at *P* < .05, and homogeneous subgroups share common superscripted letters.
